# Simultaneous Inhibition of mTOR-Containing Complex 1 (mTORC1) and MNK Induces Apoptosis of Cutaneous T-Cell Lymphoma (CTCL) Cells

**DOI:** 10.1371/journal.pone.0024849

**Published:** 2011-09-16

**Authors:** Michal Marzec, Xiaobin Liu, Maria Wysocka, Alain H. Rook, Niels Odum, Mariusz A. Wasik

**Affiliations:** 1 Department of Pathology and Laboratory Medicine, University of Pennsylvania, Philadelphia, Pennsylvania, United States of America; 2 Department of Dermatology, University of Pennsylvania, Philadelphia, Pennsylvania, United States of America; 3 Institute of Molecular Biology, University of Copenhagen, Copenhagen, Denmark; University of Chicago, United States of America

## Abstract

**Background:**

mTOR kinase forms the mTORC1 complex by associating with raptor and other proteins and affects a number of key cell functions. mTORC1 activates p70S6kinase 1 (p70S6K1) and inhibits 4E-binding protein 1 (4E-BP1). In turn, p70S6K1 phosphorylates a S6 protein of the 40S ribosomal subunit (S6rp) and 4E-BP1, with the latter negatively regulating eukaryotic initiation factor 4E (eIF-4E). MNK1 and MNK2 kinases phosphorylate and augment activity of eIF4E. Rapamycin and its analogs are highly specific, potent, and relatively non-toxic inhibitors of mTORC1. Although mTORC1 activation is present in many types of malignancies, rapamycin-type inhibitors shows relatively limited clinical efficacy as single agents. Initially usually indolent, CTCL displays a tendency to progress to the aggressive forms with limited response to therapy and poor prognosis. Our previous study (M. Marzec et al. 2008) has demonstrated that CTCL cells display mTORC1 activation and short-term treatment of CTCL-derived cells with rapamycin suppressed their proliferation and had little effect on the cell survival.

**Methods:**

Cells derived from CTCL were treated with mTORC1 inhibitor rapamycin and MNK inhibitor and evaluated for inhibition of the mTORC1 signaling pathway and cell growth and survival.

**Results:**

Whereas the treatment with rapamycin persistently inhibited mTORC1 signaling, it suppressed only partially the cell growth. MNK kinase mediated the eIF4E phosphorylation and inhibition or depletion of MNK markedly suppressed proliferation of the CTCL cells when combined with the rapamycin-mediated inhibition of mTORC1. While MNK inhibition alone mildly suppressed the CTCL cell growth, the combined MNK and mTORC1 inhibition totally abrogated the growth. Similarly, MNK inhibitor alone displayed a minimal pro-apoptotic effect; in combination with rapamycin it triggered profound cell apoptosis.

**Conclusions:**

These findings indicate that the combined inhibition of mTORC1 and MNK may prove beneficial in the treatment of CTCL and other malignancies.

## Introduction

mTOR (mammalian target of rapamycin) is a ubiquitously expressed serine/threonine kinase. mTOR associates with either protein called raptor or another named rictor and other proteins to form the mTORC1 and mTORC2 complexes, respectively. The function and signaling pathways activated by mTORC1 have thus far been much better characterized [1], [2]. Accordingly, TORC1 affects a number of key cell functions such as cell size, proliferation, protein synthesis, and angiogenesis. mTORC1 acts by phosphorylating and activating p70S6kinase 1 (p70S6K1) and inhibiting 4E-binding protein 1 (4E-BP1). p70S6K1 is a serine/threonine kinase that phosphorylates a S6 protein of the 40S ribosomal subunit (S6rp) at several sites including serines 235 and 236. In turn, 4E-BP1 is a translational repressor that negatively regulates eukaryotic initiation factor 4E (eIF-4E). Two related kinases MNK1 and, to the lesser degree, MNK2 phosphorylate eIF4E at serine 209 (S209) augmenting its activity [3]. Rapamycin and its analogs are highly specific, potent, and relatively non-toxic inhibitors of mTORC1 [1], [2].

CTCL is the most frequent type of T-cell lymphoma. Although initially usually indolent, it displays a tendency to progress to the aggressive forms with limited response to therapy and poor prognosis [4]. Sezary Syndrome (SS) is a leukemic form of CTCL in which the malignant (Sezary) T cells sometimes comprise a vast majority of the peripheral blood lymphocytes. Our recent study has demonstrated that CTCL cells display mTORC1 activation in the lymphoma stage-related fashion with the highest percentage of positive cells identified at the late, clinically aggressive stage of the large cell transformation [5]. Short-term treatment of CTCL-derived cells with the mTORC1 inhibitor rapamycin partially suppressed the cell proliferation and had little effect on their survival [5].

## Materials and Methods

### CTCL cell lines and primary cells

The MyLa2059 and MyLa3675 derived from skin lesions of advanced CTCL and the IL-2-dependent Sez-4 cell line was derived from peripheral blood, leukemic (Sezary) CTCL cells [5]. The leukemic cells used in the study were from CTCL patients with a high lymphocytosis and were >90% pure as determined by the CD4∶CD8 ratio and CD7 and/or CD26 loss by the CD4+ T cells. Cell lines and primary malignant cells were cultured at 37°C and 5% CO_2_ in RPMI 1640 medium supplemented with 10% FBS, 1% penicillin/streptomycin/Fungizone mixture, and 2 mM L-glutamine at 37°C and, in the case of Sez-4 cells, 100 U/mL of IL-2. To obtain primed cells, leukemic CTCL cells were cultured for 7 days in the presence of a mitogen PHA-L (Sigma-Aldrich, St Louis, MO) used at 10 µg/mL.

### Kinase Inhibitors

Inhibitors of MNK (MNKi) and mTORC1 (rapamycin) were purchased from Calbiochem and used at the indicated doses. MNK inhibitor, 4-Amino-5-(4-fluoroanilino)-pyrazolo[3,4-d]pyrimidine, inhibits MNK1 with IC 50 of 2.2 µM in vitro and 3 µM in vivo. It has no inhibitory activity against p38, JNK1, ERK1/2, PKC, or Src-like kinases.

### Western blot

The cells were washed in phosphate-buffered saline (PBS), centrifuged and lysed in radioimmunoprecipitation assay buffer supplemented with 0.5 mM phenylmethylsulfonyl fluoride, phosphatase inhibitor cocktails I and II from Sigma (St Louis, MO, USA) and protease inhibitor cocktail from Roche (Basel, Switzerland) as described previously [5], [6]. For normalization of gel loading, the protein extracts were assayed using the Lowry method (Bio-Rad, Hercules, CA, USA). Typically, 5–50 mg of the protein per lane was loaded. To examine protein phosphorylation, the membranes were incubated overnight with antibodies specific for S6rp S235/236, eIF4E S209, 4E-BP1 T37/46, 4E-BP1 T70, MNK1, MNK1 T197/202, MCL-1, and BcL-xL (Cell Signaling) and actin (Santa Cruz). Next, the membranes were incubated with the appropriate secondary, peroxidase-conjugated antibodies. The blots were developed using the ECL Plus System from Amersham.

### siRNA Assay

Mixture of four siRNA specific for MNK 1 and 2 oreIF4E or non-targeting siRNA (all purchased from Dharmacon) was introduced into cells at 1 µM by co-incubation in transfection media (Dharmacon Acell) for 48 h. The cells were cultured for additional 24 h, harvested and extend of the protein knock-down was examined by Western blot and RT-PCR.

### Cell proliferation (BrdU incorporation) assay

After cell culture for 1 to 10 days in the presence of inhibitors or siRNA, cell proliferation was evaluated in bromodeoxyuridine (BrdU) incorporation assay using the commercially available kit Cell Proliferation enzyme-linked immunoabsorbent assay (ELISA; Roche) according to the manufacturer's protocol. In brief, cells were seeded in 96-well plates (Corning, Corning, NY) at a concentration of 10^4^ cells/well in RPMI medium supplemented with 10% FBS and labeled with BrdU (Roche) for 4 hours. After the plate centrifugation (10 minutes at 300 g), supernatant removal, and plate drying, the cells were fixed, and the DNA was denaturated by the addition of 200 mL FixDenat reagent. The amount of incorporated BrdU was determined by incubation with a specific antibody conjugated with peroxidase followed by colorimetric conversion of the substrate and OD evaluation using the ELISA plate reader.

### Cell Growth: Proliferation and Survival (MTT Enzymatic Conversion) Assay

Cell lines were seeded in 96-well plates at 1×10^4^ cells/well in RPMI medium supplemented with 10% FBS. After 6 h culture, the cells were exposed in triplicates to serial dilutions of the inhibitors. After 1–14 days, the relative number of viable cells was determined by the use of MTT reduction colorimetric assay (Promega).

### Cell apoptosis (terminal dUTP nick-end labeling: tunel) assay

We used the ApoAlert DNA Fragmentation Assay Kit from BD Biosciences (San Jose, CA) according to the manufacturer's protocol. In brief, cells were cultured at 0.5×10^6^ cells/mL for 3, 7 or 14 days with inhibitors. The cells were collected, washed twice in PBS, and fixed with 1% formaldehyde/PBS. After the wash, cells were permeabilized with 70% ice-cold ethanol for at least 2 hours, washed, and incubated in TdT incubation buffer for 1 hour at 37°C. The reaction was stopped by adding 20 mM EDTA, and the cells were washed twice in 0.1% Triton X 100/BSA/PBS. Finally, samples were resuspended in 0.5 mL of PI/RNAse/PBS, collected, and analyzed by flow cytometry (FACSort; Becton Dickinson, Franklin Lakes, NJ) using the CellQuest PRO software.

### Statistics

The significance of difference between controls and different treatment conditions in BrdU, MTT and terminal dUTP labeling assay was evaluated using Student's t-test. P value of <0.05 was considered to be statistically significant. All presented results are calculated as mean +/− S.D. of three or four separate experiments.

## Results

### Rapamycin partially inhibits growth of CTCL cells and promotes eIF4E phosphorylation at serine 209

To evaluate impact of the extended exposure of malignant T cells to mTORC1 inhibition, we treated two CTCL-derived cell lines, MyLa2059 and MyLa3675, with rapamycin for up to 10 days. As shown in Fig. 1A, rapamycin, used at the predetermined saturating dose [5] was able to suppress CTCL cell proliferation as determined by the BrdU incorporation assay (p<0.05 for days 2–10 as compared to the untreated control). However, the suppression was only partial despite the very effective and persistent inhibition of the mTORC1 signaling as determined by the marked, sustained dephosphorylation of S6rp and 4E-BP1 with the latter dephophorylation appearing less pronounced in MyLa2059 (Fig. 1B). . Of note, mTORC1 inhibition enhanced phosphorylation of eIF4E at S209 (Fig. 1B) suggesting that phospho-eIF4E may be involved in supporting the residual cell growth.

**Figure 1:** Rapamycin partially inhibits proliferation of T-cell lymphoma cells and promotes eIF4E S209 phosphorylation. The CTCL-derived cell lines MyLa2059 and MyLa3675 were treated in triplicates with 200 nM of rapamycin (mTORC1i) for up to 10 days and (A) labeled with BrdU for the last 4 hr of the culture and examined using the EIA plate reader (the result shows mean value of four separate experiments) or (B) lysed and analyzed by Western blotting with antibodies against the depicted phosphorylated and total proteins with detection of actin serving as the loading control.

### MNK mediates eIF4E S209 phosphorylation

Because MNK 1 and 2 kinases have been reported to target the eIF4E S209 site [3], [7], we examined next the effect of MNK inhibition on the eIF4E S209 phosphorylation status. A selective, small molecule MNK inhibitor profoundly suppressed eIF4E S209 phosphorylation in the dose-dependent manner without affecting phosphorylation of Akt-T308, used as control of the inhibitor's specificity (Fig. 2A). The inhibitor suppressed not only the spontaneous, but also the rapamycin-enhanced eIF4E S209 phosphorylation (Fig. 2B), indicating that MNK1/2 is the sole kinase of the S209 site responsible for its baseline as well as the mTORC1 inhibition-augmented phosphorylation. MNK phosphorylation at T197/202 as well as the expression of two anti-apoptotic proteins MCL-1 and BcL-xL remained unaffected indicating that MNK does not self-phosphorylate itself at this key site, on one hand, and that MCL-1 and BcL-xL are not affected by the MNK and mTORC1 inhibition in the CTCL cells. To confirm the MNK's role in the eIF4E S209 phosphorylation, we inhibited MNK expression using siRNA active against both MNK1 and MNK2. The MNK1/2 depletion resulted in the proportionate decrease in the amount of S209-phosphorylated eIF4E protein that matched the decrease achieved by the depletion of eIF4E itself using the eIF4E-specific siRNA (Fig. 2C).

**Figure 2:** MNK inhibition suppresses eIF4E S209 phosphorylation. A: effect of MNK1/2 inhibitor (MNKi) used at various concentrations on eIF4E S209 phosphorylation in MyLa2059 and MyLa3675 cell lines with Akt T308 phosphorylation serving as a control. B: effect of simultaneous application of MNKi (5 µM) and mTORC1i (200 nM) on phosphorylation of eIF4E S209, S6rp S235/236, and MNK T197/202 and expression of the anti-apoptotic proteins Mcl-1 and BcL-xL. C: effect of siRNA-mediated MNK1 and MNK2 depletion on eIF4E S209 phosphorylation in the presence or absence of rapamycin. D: effect of simultaneous exposure of IL-2-dependent CTCL cell line Sez-4 to MNKi and mTORC1i on phosphorylation and expression the depicted proteins. E: effect of simultaneous treatment of patient-derived, primed Sezary CTCL cells to MNKi and mTORC1i on phosphorylation and expression the depicted proteins.

To determine if eIF4E is phosphorylated by MNK also in other types of CTCL cells, we examined leukemic (Sezary) cells, both in the form of an established IL-2-dependent cell line Sez-4 and primary cells from two CTCL patients. Our previous study [5] has established that, in contrast to the CTCL cell lines and tissues, native leukemic CTCL cells are quiescent and require both mitogen priming and IL-2 stimulation to activate mTORC1 as well as PI3K/Akt and MEK/ERK signaling pathways. As shown in Fig. 2D, Sez-4 cell line displayed essentially the same pattern of response to mTORC1 and/or MNK inhibition as MyLa2059 and MyLa3675 cells, including the inhibition of eIF4E S209 phosphorylation by the MNK inhibitor and enhancement of this phosphorylation secondary to mTORC1 inhibition. While the native leukemic CTCL also displayed eIF4E S209 phosphorylation that was suppressed by the MNK inhibitor (Fig. 2E), the rapamycin-induced enhancement of the phosphorylation was not definitive, mostly likely reflecting overall less malignant phenotype of these cells. Regardless, the presence of the MNK-mediated eIF4E phosphorylation in all types of CTCL cells examined, strongly suggests that it may contribute to their malignant phenotype.

### eIF4E S209 phosphorylation is independent of MEK, p38 MAPK, PKC, PKA, and PI3K

Previous studies have implicated MEK1/2-ERK1/2 and p38 MAPK-MSK pathways, separately and in combination in MNK activation in some cell systems [8]. However, inhibition of MEK1/2, p38 MAPK (separately or in combination), PKC, PKA (Fig. 3A) or PI3K (Fig. 3B) did not suppress eIF4E phosphorylation indicating involvement of a different kinase that remains to be identified. Of note, activation of MNK independent of ERK1/2 and p38 MAPK has also been described by others [8].

**Figure 3:** Lack of effect on eIF4E phosphorylation of several kinase inhibitors. A and B: Expression of eIF4E S209 was examined after treatment of MyLa 2059 cells with inhibitor of p38 MAPK, MEK1/2 (U0126), PKC (Go6983), PKA (Bisindolylmaleimide I) and PI3K (Wortmannin and LY294002). Expression of phospho-Akt T308 and -ERK1/2 T202/Y204 and actin and cell treatment with MNKi served as controls.

### Inhibition of MNK suppresses growth of CTCL cells

To determine if MNK controls proliferation of CTCL cells, we treated MyLa2059 and MyLa3675 cells with the MNK inhibitor, applied either as a single compound or together with rapamycin. While MNK inhibition alone suppressed the BrdU uptake, this effect was more pronounced in the presence of rapamycin indicating an additive effect of the compounds (Fig. 4A). Similarly, combination of the siRNA-mediated MNK depletion and rapamycin resulted in the decreased CTCL cell proliferation (Fig. 4B). Of note, siRNA-triggered depletion of eIF4E markedly affected the BrdU uptake, in particular when applied jointly with rapamycin, highlighting the importance of eIF4E in promoting cell proliferation.

**Figure 4:** Simultaneous mTORC1 and MNK inhibition suppresses growth and induces apoptosis of CTCL-derived cells.

### Combined inhibition of mTORC1 and MNK induces apoptotic cell death of CTCL cells

To determine if MNK affect long-term growth of CTCL cells, we exposed MyLa2059 and MyLa3675 cells for up to 14 days to the MNK inhibitor in the presence or absence of rapamycin (Fig. 4C). While each of the drugs alone exerted a moderate (rapamycin: p<0.05 as compared to the control) or mild (MNKi) inhibitory effect on the cell growth as determined by the MTT enzymatic conversion, their combination profoundly affected the growth in the time-dependent manner (p<0.01 vs. control). As shown in Fig. 4D, the leukemic cells from two CTCL patients yielded very similar result (p<0.01) further supporting the notion that the mTORC1 and MNK inhibitor combination may be therapeutically effective.

To directly examine MNK effect on the cell survival, we performed the DNA fragmentation (tunel) assay in the MNK inhibitor- and/or rapamycin-treated MyLa2059 and MyLa3675 cells. Whereas MNK inhibitor alone induced very limited cell death, its combination with rapamycin resulted in profound apoptosis of the CTCL cells (Fig. 4E; p<0.01 at day 7 and 14 vs. control).

## Discussion

Given the critical role of mTORC1 signaling in cell biology and carcinogenesis as well as the availability of very potent and highly specific mTORC1 inhibitors from the rapamycin family, there has been an immense interest in inhibiting the pathway in patients with various malignancies and other ailments [1]. In fact, numerous clinical trials have been conducted with mTORC1 inhibitors in the large spectrum of cancer types [1], [9]. The drugs used as single agents showed substantial efficacy in several different tumors including transplant-associated lymphoma [10], [11] and Kaposi sarcoma [12], [13], tuberous sclerosis-related astrocytoma [14], and mantle cell and other non-Hodgkin lymphomas [15]. Recently, two mTORC1 inhibitors gained FDA approval for treatment of the renal cell carcinoma [16], [17]. However, the treatment with rapamycin-type compounds typically leads to the clinically stable disease or partial remission rather than the tumor elimination [9]. This suboptimal drug effect is likely due at least in part to the cytostatic rather than cytotoxic properties of the mTORC1 inhibitors. Therefore, there is a great need for the drug combination therapy that ideally would result in the complete remissions and cancer cures. However, most of the attempts to combine mTORC1 inhibitors with other drugs, typically the standard chemotherapeutic agents targeting DNA replication, have so far been rather disappointing, on occasion leading to the drug antagonism, although some combinations, e.g. with cis-platin [18] or methotrexate [19] seem promising based on the preclinical studies.

Here we report that the extended exposure of CTCL cells to the combination of mTORC1 and MNK inhibitors essentially abolishes the cell growth by triggering extensive apoptotic cell death. MNK inhibition eliminates S209 phosphorylation of the indirect target mTORC1 target eIF4E, not only basal but also rapamycin-enhanced, the latter noted in CTCL cell lines. Although we cannot exclude that other MNK targets unrelated directly to the protein synthesis also contribute to cell survival, several observations indicate that the effect of MNK on the eIF4E-containing complex and protein translation are critical in this regard. First, MNK inhibition alone has very little effect on the cell viability; only the combined inhibition of MNK and mTORC1 triggers the apoptosis. Second, recent studies indicate that the inhibition of the eIF4E complex by mTORC1 inhibitors is incomplete due to the relatively ineffective suppression of the 4E-BP1 phosphorylation [20]. The addition of MNK inhibitor appears to correct this deficiency and the MNK-mTORC1 inhibitor combination fully inhibits eIF4E leading to not only suppression of CTCL cell proliferation but, strikingly, also to induction of cell death. The study by Furic et al. [21] showed that the substitution in eIF4E of serine with alanine at position 209 (S209A) inhibited the development of prostatic carcinoma initiated by the prostate-specific loss of PTEN. This finding supports the notion that the MNK-mediated eIF4E S209 phosphorylation plays a key role in the biology of malignant cells, although MNK seems to modify also other members of the translation initiation complex [8], [22]. Finally, the other key MNK targets such as hnRNP A1 and Spry2 are involved in generating anti-growth signals by inducing expression of TNFa and enhancing ERK signaling, respectively. Therefore, their inhibition should not induce cell apoptosis. However, the specific proteins responsible for initiating the apoptosis induced by the joint mTORC1-MNK inhibition remain to be identified. Although MCL-1 expression has been reported as translationally regulated by mTORC1 and MNK in some cell types [7], inhibition of neither of them affected expression of MCL-1 and of another anti-apoptotic protein BcL-xL (Fig. 2). Regardless, our findings strongly suggest that the simultaneous inhibition of mTORC1 and MNK1/2 kinases, both targeting eIF4E activity, may prove highly efficacious in treatment of CTCL and, in all likelihood, many other malignancies. Furthermore, since mTORC1 is activated by a large spectrum of oncogenic cell-surface receptors and intracellular kinases [1], combined inhibition of MNK and the relevant oncogenic kinase upstream of mTORC1 may also prove therapeutically beneficial. The highly effective combination of BCR-ABL inhibitor with MNK inhibitor [23], suggests that this indeed may be the case.
